The article "The Diagnostic Value of GGT-Based Biochemical Indicators for Choledocholithiasis with Negative Imaging Results of Magnetic Resonance Cholangiopancreatography" was published in 2022. Journal: Contrast Media Mol Imaging.

# The Diagnostic Value of GGT-Based Biochemical Indicators for Choledocholithiasis with Negative Imaging Results of Magnetic Resonance Cholangiopancreatography

**DOI:** 10.1155/2022/7737610

**Published:** 2022-06-27

**Authors:** Huajun Lin, Xiaona Zhou, Zhongtao Zhang

**Affiliations:** Department of General Surgery, Beijing Friendship Hospital, Capital Medical University and National Clinical Research Center for Digestive Diseases, Beijing 100050, China

## Abstract

To reveal the relationship between a group of preoperative biochemical indicators such as GGT, ALP, ALT, AST, TB, and DB and the occurrence of common bile duct stones in patients with negative results of magnetic resonance cholangiopancreatography, a retrospective diagnostic accuracy clinical test is conducted in this study. In order to reduce the missed diagnosis rate of choledocholithiasis and perform more accurate common bile duct exploration, 466 patients who underwent surgical treatment of cholelithiasis from January 2014 to December 2015 have been analyzed retrospectively. Firstly, the confounding factors are corrected through Binary Logistic regression. Then, the diagnostic efficacy of each indicator is measured by the ROC curve among different types of patients. In all patients, the top three individual indicators with the greatest AUC curve area for predicting common bile duct stones can be observed from the results of MRCP, *γ*-glutamyl transpeptidase, and alkaline phosphatase. Besides, the diagnostic efficiency of the comprehensive evaluation is higher than that of all individual indicators. For MRCP-negative patients, the top three largest AUC curve area of the diagnostic efficacy for choledocholithiasis were GGT, ALP, and DB. For patients who have a suspected diagnosis of secondary choledocholithiasis, the diagnostic efficacy of the combination of imaging results, biochemical indexes, common bile duct width, and other abnormal indicators for choledocholithiasis is much higher than that of the single abnormal biochemical indexes for the prediction of choledocholithiasis. For MRCP-negative patients, GGT, ALP, DB, and the width of common bile duct diameter are valuable for the prediction of common bile duct stones, and GGT is the most valuable diagnostic predictor.

## 1. Introduction

Cholelithiasis is a common and frequently occurring disease worldwide. Simple gallbladder stones are the main component of cholelithiasis, and approximately 10%–30% of gallstone patients also suffer from choledocholithiasis [1, 2]. For gallbladder stones combined with symptomatic common bile duct stones, the clinician can easily confirm the diagnosis preoperatively. However, some patients with cholecystolithiasis combined with choledocholithiasis are easily missed by clinicians due to asymptomatic choledocholithiasis [3]. If these patients only undergo laparoscopic cholecystectomy (LC), residual postsurgical common bile duct stones will be at risk of complications such as acute cholangitis and acute membranous adenitis [4]. Therefore, it is particularly important to investigate whether patients have cholecystolithiasis combined with choledocholithiasis before operation. For the treatment of secondary choledocholithiasis, the safety and effectiveness of the “one-step approach”, namely, the combination of laparoscopic cholecystectomy and choledochoscopic choledocholithotomy, have been confirmed [5, 6]. Most diagnoses of common bile duct stones mainly relied on traditional common bile duct exploration indicators including the diameter of the common bile duct (greater than or equal to 0.8 cm), abdominal ultrasound scan, patient's history of biliary pancreatitis, and multiple small gallbladder stones or gallbladder neck stones previously. With the development of imaging technology, magnetic resonance cholangiopancreatography (MRCP) has been reported to have great value in the diagnosis of choledocholithiasis. Studies suggest that an abdominal ultrasound scan is the primary investigative modality for cholelithiasis [7]. However, MRCP is used for further examination of common bile duct stones. Although MRCP has relatively high accuracy, it cannot screen out all common bile duct stones. The reason is that there are a large number of patients with cholelithiasis, whether the traditional assessment of common bile duct stones or the MRCP examination [8]. It should be noted that some patients with choledocholithiasis will be missed and misdiagnosed. Besides, not all hospitals at all levels have MRI machines that can complete MRCP examinations. A certain proportion of patients can not routinely undergo MRCP examination before an operation, such as patients after partial coronary stent implantation, orthopedic prosthesis implantation, contraceptive ring implantation, etc. Thus, plenty of patients with cholelithiasis will be misdiagnosed or misdiagnosed regardless of the traditional methods for assessing choledocholithiasis or MRCP examination.

In the routine clinical work, we found that patients with asymptomatic secondary choledocholithiasis often had abnormal liver function indicators, which may have predictive value for asymptomatic secondary choledocholithiasis. Therefore, the preoperative biochemical indicators, preoperative imaging results, and surgical outcomes of patients who underwent laparoscopic cholecystectomy and choledochoscopic exploration in our hospital were retrospectively analyzed. In addition, a clinical trial study was conducted on the diagnostic accuracy to analyze the correlation of each index with common bile duct stones. Particularly, the diagnostic efficacy of each biochemical indicator of common bile duct stones in MRCP-negative patients with normal width of the common bile duct was the main focus of the study. The diagnostic efficacy of blood biochemical parameters in MRCP-negative choledocholithiasis was summarized and analyzed to provide clinical evidence for the preoperative diagnosis of secondary choledocholithiasis in patients with negative imaging.

## 2. Related Work

Cholelithiasis is a common disease of the digestive system. Choledocholithiasis (CBDS) is estimated to be present in 10–20% of individuals with symptomatic gallstones [9]. A study has suggested an upward trend in the incidence of cholelithiasis and morbidity due to this disease in younger individuals, which may be mainly related to factors such as lack of exercise, obesity, diabetes, and early pregnancy [10]. Cholelithiasis is divided into intrahepatic bile duct stones and extrahepatic bile duct stones according to anatomical location [11]. Common bile duct stones can be classified into primary and secondary types. Some secondary common bile duct stones are often those that traverse to the bile duct from the gallbladder with bile excretion via the cystic duct. As some of the stones float in the common bile duct, there will be no clinical manifestations associated with biliary obstruction or stone impaction. Small stones or sediment-like biliary sludge deposits in the common bile duct can only be detected by intraoperative biliary exploration [12]. Sometimes the presence of small calculi was missed in preoperative examination, so that the surgeon did not carry out effective exploration of the common bile duct during the operation, resulting in residual common bile duct calculi. Common bile duct exploration should also not be performed too aggressively, as common bile duct exploration can lead to some of the more serious complications [13]. Therefore, the assessment and management of choledocholithiasis should be precise and cautious [14]. Generally, surgeons rely on traditional indications for common bile duct exploration to evaluate patients for possible common bile duct stones or to decide whether intraoperative biliary exploration should be performed. These indications include the following: common bile duct width > 8 mm; a medical history of biliary pancreatitis; imaging suggestive of common bile duct stones; multiple small gallbladder stones; intraoperative palpable common bile duct stones; intraoperative cholangiography suggestive of common bile duct stones; and preoperative ERCP results suggestive of common bile duct stones [15, 16]. With the development of medical technologies, new biochemical and imaging indicators have been applied to predict common bile duct stones. Through the invention and development of MRCP, intraoperative cholangiography and diagnostic ERCP have been gradually replaced and MRCP plays an increasingly important role in the diagnosis of common bile duct calculi detection [17, 18]. However, due to the relatively expensive cost of MRCP, it is not ideal from a health economics perspective if MRCP is routinely performed on every patient with choledocholithiasis, which will prolong the patient's hospital stay and increase the financial burden. Moreover, the hardware requirements of MRCP, a special biliary imaging examination, are not met by all levels of hospitals, and some patients have relative contraindications to MRCP. For patients who are unable to undergo MRCP or have negative MRCP results, the preoperative evaluation of choledocholithiasis relies on the remaining laboratory tests and imaging studies; however, there is no clear guideline as to whether all of these multiple assessment criteria should be considered comprehensively or whether it is better to focus on a single indicator.

GGT is a cell surface enzyme associated with GSH metabolism and plays an important role in cellular metabolism against oxidative stress; accordingly, GGT can regulate redox-sensitive functions such as antioxidant defense, cell proliferation, and apoptosis homeostasis [19, 20]. GGT plays an important role in oxidative stress by converting glutathione to cysteine, glutamate, and glycine in cellular metabolism. Because cysteine is essential for intracellular glutathione (a major antioxidant) synthesis, GGT concentration can reflect the degree of oxidative stress in tissue cells [21, 22]. Serum GGT has been shown to be correlated with the metastasis and prognosis of various malignancies [23, 24] and is closely associated with the efficacy and neurotoxic side effects of chemotherapeutic agents in malignant tumors [25–27]. It is still a classical biochemical index studied by a wide range of researchers.

GGT is distributed in all organs of the body, with a higher concentration in the biliary epithelium. It is closely related to the occurrence and development of various diseases [28–31]. In the diagnosis and treatment of biliary-related diseases, especially cholelithiasis, GGT has always been a popular biochemical indicator [32]. Cholelithiasis is a common benign biliary tract disease, with its pathological process leading to biliary tract injury and changes in various metabolic enzymes in bile duct epithelial cells, among which GGT, ALP, and other liver enzymatic indicators have auxiliary diagnostic values for choledochal stones with obstructive jaundice [33]. However, few studies have been reported on the predictive value of this type of choledocholithiasis with negative imaging results.

Based on these results, the authors conducted a retrospective case-control designed clinical trial for diagnostic accuracy, which suggested that the overall index (combined MRCP results, common bile duct diameter, and GGT, ALP, TB, DB, ALT, and AST results) is more effective than all individual indexes for the diagnosis of common bile duct stones in patients who underwent common bile duct exploration. In patients with negative MRCP results, there was no statistically significant difference between the diagnostic efficacy of the overall index and that of the GGT index alone for the diagnosis of common bile duct stones. In patients with negative MRCP results and a nonwide diameter of the common bile duct, the diagnostic efficacy of the overall indexes of GGT, ALP, TB, DB, ALT, and AST was not superior to that of the individual indexes of GGT, ALP, and ALT for the diagnosis of common bile duct stones.

In patients with negative MRCP results, the biochemical parameters GGT, ALP, and DB, and the width of the common bile duct diameter are valuable for predicting common bile duct stones, among which the diagnostic efficacy of GGT is particularly significant, which may be due to the higher concentration of GGT in the bile duct epithelium. When the stones are not large enough to be visualized on imaging, there are still kinetic changes of biliary sludge in the bile duct. When bile is accumulating, the countercurrent hydrostatic pressure will cause acute damage to the bile duct and bile duct epithelium, as well as the solubilizing effect of the bile acids on hepatocyte membrane-bound enzymes, resulting in elevated serum GGT, which is the reason why elevated GGT caused by the increase in bile duct pressure in the early stage of choledocholithiasis is prior to the increase in serum bilirubin. In patients with negative MRCP results, once the preoperative GGT index is found to be higher than the critical value, the patient should be highly suspected of having common bile duct stones, and LCTCBDE should be performed intraoperatively if possible. If intraoperative common bile duct exploration is not performed, the patient should be closely observed and followed up after surgery. ERCP and other biliary tract-related imaging examinations should be reviewed in a timely manner to avoid missing diagnosis. The common bile duct width for the determination of common bile duct stones has only a certain diagnostic efficacy in patients with negative MRCP results, probably due to the small size of the common bile duct stones that merely float in the common bile duct and do not block the bile outflow tract to a high degree, which leads to the unobvious widening degree of the common bile duct. The diameter of the common bile duct is commonly assessed using ultrasound. However, due to the deep location of the common bile duct and its susceptibility to intestinal gas interference, the assessment of the diameter of the common bile duct is relatively limited and the resulting predicted value is not accurate. In other cases, the common bile duct is widened only after a transient obstruction by bile duct stones that are discharged into the duodenum by biliary contraction regulation, and then the residual small stones in the common bile duct do not widen the common bile duct significantly.

## 3. Methodology

### 3.1. Experimental Design and Population

This study is a retrospective case-control clinical trial of diagnostic accuracy. After the initial screening using the following inclusion criteria: (1) males and females aged >18 years; (2) elective surgical treatment for cholelithiasis at our hospital; and (3) complete preoperative routine blood and biochemical C21 results and exclusion criteria: (1) age <18 years; (2) patients without preoperative C21 biochemical index results; (3) patients unable to cooperate with the study of cancer or AIDS; and (4) pregnant and lactating women, we obtained data from 514 consecutive patients who underwent surgical treatment for cholelithiasis in our department between January 2014 and December 2015. We obtained data, including medical record number, age, sex, and preoperative biochemical indices. Alanine transaminase (ALT), Aspartate aminotransferase (AST), Alkaline phosphatase (ALP), Gamma-glutamyl transpeptidase (GGT), total bilirubin (TB), direct bilirubin (DB), amylase (AMY), ultrasound results, common bile duct diameter, MRCP results, CT results, primary diagnosis, comorbid diagnoses, name of primary surgery, and names of other surgical operations were also obtained. The formed calculi were clearly found during LCBDE as the “golden standard” of choledocholithiasis.

### 3.2. Observational Biochemical Indicators and Imageology

All patients had undergone the biochemical c21-included blood tests within one week before the operation. The standard values of biochemical indexes were based on our biochemical C21 indexes, *i*. e. AST > 40 U/L, ALT > 50 U/L, GGT > 45 U/L, ALP > 125 U/L, TB > 17.1 *µ*mol/L, and DB > 6.8 *µ*mol/L. Each biochemical index was strictly calibrated and entered, and was measured according to the same standard as our hospital [7]. A majority of the 349 patients (349/466) had undergone MRCP examination before surgery. The MRCP report described the evaluation of common bile duct stones as definite common bile duct stones, possible common bile duct stones, and no evidence of the presence of common bile duct stones. The cases with the former two descriptions in MRCP's result (definite common bile duct stones or possible common bile duct stones) were defined as MRCP-positive (presence of common bile duct stones) and those with the latter were defined as MRCP-negative (imaging not considered the presence of common bile duct stones). A total of 95 patients had preoperative abdominal ultrasound reports describing whether they had possible common bile duct stones. Based on the MRCP or abdominal ultrasound imaging reports, values for imaging common bile duct diameter were included in the assessment of 450 patients.

### 3.3. Mode of Surgery

All patients underwent a surgical-focused treatment plan involving laparoscopic cholecystectomy + laparoscopic transcystic common bile duct exploration (LC + LCTCBDE), choledochotomy + laparoscopic transcystic common bile duct exploration (non-LC + LCTCBDE), choledochoscopic lithotripsy, and LCBDE converted to laparotomy. Each patient was operated on by a team of skilled surgeons with comparable surgical experience [8]. We defined laparoscopic cholecystectomy + laparoscopic transcystic common bile duct exploration as LC + LCTCBDE and the rest of the procedures as non-LC + LCTCBDE when performing subsequent statistical classification.

The data were analyzed according to the objective results of surgical exploration and the results of various laboratory indicators. All patients provided written informed consent, and the study was approved by the Ethics Committee of Beijing Friendship Hospital (No. 2018-P2-028-01).

### 3.4. Statistical Methods

In this study, the basic data of patients were compared between the two groups using the *t*-test and chi-square test using the statistical software SPSS 22.0. For assessment of diagnostic efficacy, the corrected predictive probability of each indicator for common bile duct stones was obtained by incorporating confounding factors and performing multivariate binary logistic regression for each individual indicator. Thereafter, sensitivity, specificity, and area under the curve were calculated from this corrected predictive probability. The AUC difference, *z* value, and *p* value between each individual indicator and all the indicators were obtained by plotting the corrected ROC curves and *z*-test between groups using the MedCalc software. *p* values < 0.05 were considered statistically significant.

## 4. Results

### 4.1. Baseline Characteristics

According to the inclusion and exclusion criteria, we first entered the basic information of 514 patients and further collated the data to exclude 48 patients, including 8 with MIRRIZI syndrome, 9 with combined intrahepatic bile duct stones, 5 with combined chronic liver disease, 7 with diagnosed gallbladder malignancy, and 19 with incomplete recorded data. Lastly, 466 patients were included in this study, of which 398 patients were <75 years old and 68 were ≥75 years old. Of 198 and 268 male and female patients, respectively, 448 had LC + LTCBDE and 18 had non-LCTCBDE (2 intermediate open, 14 choledochotomy stone extraction, 2 choledochoscopic lithotripsy). Further, 349 patients had definitive imaging findings reported by MRCP completed preoperatively. The specific width of the common bile duct assessed was reported in preoperative imaging (ultrasound, CT, MRCP) in 250 patients, and all patients had undergone preoperative biochemical markers containing ALT, AST, ALP, GGT, TB, and DB. A total of 315 patients were diagnosed with common bile duct stones during surgery, and 151 patients were not found to have common bile duct stones during surgery. As the blood amylase test and abdominal computed tomography (CT) are not routinely performed before laparoscopic cholecystectomy + common bile duct exploration in our institution, only 64 patients included in this study had results of a preoperative blood amylase concentration test, and 36 had results of the preoperative plain/enhanced CT of the abdomen.  Table 1 shows the baseline characteristics of all patients. LC + LCTCBDE represents laparoscopic cholecystectomy + laparoscopic transcystic common bile duct exploration. Non-LC + LCTCBDE represents choledochotomy + laparoscopic transcystic common bile duct exploration, choledochoscopic lithotripsy, and LCBDE converted to laparotomy. The *t*-test was used to analyze the differences between groups for continuous variables, and the chi-square test for differences between the groups for categorical variables. We defined *p*-value < 0.05 as statistically significant.

### 4.2. Assessment of the Diagnostic Efficacy of All Indicators for Common Bile Duct Stones

In all patients, the ROC curve of diagnostic efficacy of each indicator for common bile duct stones after correction found sensitivity, specificity, and AUC of 76.11%, 86.6%, and 0.872, respectively, on combined assessment of all factors for common bile duct stones. The top three individual indicators with the largest AUC for the diagnostic efficacy of common bile duct stones were MRCP (with an AUC of 0.804, sensitivity of 70.63%, and specificity of 87.63%), GGT (AUC of 0.761, sensitivity of 78.1%, and specificity of 63.58%), and ALP (AUC of 0.753, sensitivity of 60.0%, and specificity of 85.43%). However, the diagnostic efficacy of the combined assessment of all factors was higher than that for individual factors. There was a statistically significant difference between the ROC curves of the all-factor composite assessment and the confounding factors (baseline) (AUC difference of 0.259, *z* value 7.532, *p* < 0.0001). A statistically significant difference was seen between the ROC curves of the all-factor composite assessment and MRCP (AUC difference of 0.0658, *z* value 3.716, *p* = 0.0002). In addition, statistically significant differences were found between the ROC curves for the all-factor composite assessment and CBDD (AUC difference of 0.117, *z* value 5.287, *p* < 0.0001). Statistically significant differences were also found between the ROC curves of the all-factor composite assessment and GGT (AUC difference of 0.0987, *z* value 4.587, *p* < 0.0001). *p* < 0.0001).  Table 2 illustrates the diagnostic efficacy of the predictors for common bile duct in all patients. In addition, Figure 1 shows the comparison of receiver operating characteristic curves between total indicators and individual indicators. The difference value of each area under the curve (ΔAUC) can be observed, and the *z*-test is used for statistical comparison between the groups. The *p* value less than 0.05 is considered statistically significant. The corrected predictive probability of each indicator for common bile duct stones was obtained by including confounding factors, performing multivariate binary logistic regression with each individual indicator, and calculating the sensitivity, specificity, and area under the curve from this corrected predictive probability. *p* value < 0.05 was defined as statistically different. CBDD stands for common bile duct diameter width. Total represents an integral predictive indicator including all factors in the table.

### 4.3. Evaluation of the Diagnostic Efficacy of Each Index for Common Bile Duct Stones in MRCP-Negative Patients

Among the patients with negative MRCP results, the ROC curve of the diagnostic efficacy of each index for common bile duct stones after correction showed that the sensitivity of the combined assessment of all factors for common bile duct stones was 56.79%, the specificity was 88.24%, and the AUC was 0.759. The top three individual indexes with the largest AUC for the diagnostic efficacy of common bile duct stones were GGT (AUC of 0.704, sensitivity of 69.88%, and specificity of 68.24%), ALP (AUC of 0.701, sensitivity of 55.42%, and specificity of 85.88%), and DB (AUC of 0.652, sensitivity of 55.42%, and specificity of 76.47%). The ROC curves for the all-factor composite assessment were significantly different from those of the confounders (baseline) (AUC difference of 0.146, *z* value 3.367, *p* = 0.0008) and the ROC curves for the all-factor composite assessment were statistically significantly different from those of the ALP (AUC difference of 0.0538, *z* value 2.207, *p* = 0.0426). A statistically significant difference was noted between the ROC curves of the all-factor composite assessment and DB (AUC difference of 0.104, *z* value 2.686, *p* = 0.0072). No statistically significant difference was found between the ROC curves of the all-factor composite assessment and GGT (AUC difference of 0.052, *z* value 1.798, *p* = 0.0722). The ROC curve for the all-factor composite assessment was significantly different from CBDD (AUC difference of 0.121, *z* value 3.273, *p* = 0.0011).  Figure 2 shows the comparison of receiver operating characteristic curves between total indicators and individual indicators in the patients with negative MRCP. The difference value of each area under the curve (ΔAUC) is demonstrated, and the *z*-test was used for the statistical comparison between the groups. The *p* value less than 0.05 is considered statistically significant.  Table 3 shows the diagnostic efficacy of the predictors for common bile duct in patients with a negative result of MRCP. In addition, Figure 2 demonstrates the comparison of receiver operating characteristic curves between total indicators and individual indicators in the patients with negative MRCP.

### 4.4. Evaluation of the Diagnostic Efficacy of Each Index for Common Bile Duct Stones in Patients with Double Negative MRCP and Common Bile Duct Diameter

For the patients with negative MRCP results and common bile duct diameter <0. 8 cm, it was found that the ROC curve of the diagnostic efficacy of each index for common bile duct stones after correction showed sensitivity of 72.41%, specificity 69.74%, and AUC 0.732. The top three individual indexes of the AUC curve area of the diagnostic efficacy for common bile duct stones were: GGT (AUC of 0.715, sensitivity of 65.52%, specificity of 68.42%), ALP (AUC of 0.709, sensitivity of 63.79%, specificity of 73.68%), and ALT (AUC of 0.658, sensitivity of 50.00%, specificity of 75.00%).

The ROC curve for the all-factor composite assessment was significantly different from those of the confounders (baseline) (AUC difference of 0.142, *z* value 2.879, *p* = 0.004). The ROC curve for the all-factor composite assessment was not statistically different from the GGT (AUC difference of 0.0177, *z* value 0.722, *p* = 0.4705), and the ROC curve for the all-factor composite assessment was not statistically different from the ALP (AUC difference of 0.0236, *z* value 0.979, *p* = 0.3249). ROC curves for combined assessment of all factors were not statistically different from those of ALP (AUC difference of 0.0236, *z* value 0.984, *p* = 0.3249) and ALT (AUC difference of 0.0745, *z* value 1.774, *p* = 0.0761). The diagnostic efficacy of the predictors for common bile duct in patients with both negative results of MRCP and CBDD is listed in Table 4.  Figure 3 shows the comparison of receiver operating characteristic curves between total indicators and individual indicators in the patients with negative results of MRCP and CBDD (less than 0.8 cm).

## 5. Conclusions

In this clinical study, we suggest that in patients with suspected secondary choledocholithiasis, abnormalities in individual biochemical indexes of GGT, ALP, ALT, AST, TB, or DB cannot replace the diagnostic efficacy of multiple index abnormalities, including imaging and the width of the common bile duct. Therefore, for such patients, it is necessary to complete all the relevant laboratory tests and imaging examinations as far as possible and comprehensively evaluate various indicators to get the most accurate evaluation. For patients with negative MRCP results, GGT, ALP, and DB, and the width of the common bile duct diameter are valuable for predicting common bile duct stones, and the diagnostic efficacy of GGT is particularly significant.

## Figures and Tables

**Figure 1:** Receiver operating characteristic curves between total indicators and individual indicators: (a) total indicators and baseline data including age and sex; (b) total indicators and the result of magnetic resonance cholangiopancreatography; (c) total indicators and the diameter of the common bile duct; and (d) total indicators and serum glutamine transpeptidase level.

**Figure 2:** Receiver operating characteristic curves between total indicators and individual indicators in the patients with negative MRCP: (a) total indicators and diameter of common bile duct; (b) total indicators and the result of direct bilirubin; (c) total indicators and alkaline phosphatase levels; and (d) total indicators and serum glutamine transpeptidase levels.

**Figure 3:** Receiver operating characteristic curves between total indicators and individual indicators in the patients with negative results of MRCP and CBDD (less than 0.8 cm): (a) total indicators and baseline data including age and sex; (b) total indicators and serum glutamine transpeptidase levels; (c) total indicators and alkaline phosphatase levels; and (d) total indicators and alanine transaminase levels.

**Table 1:** Baseline characteristics of all patients.

Basic information	Total	Average value	Diagnosis of CBDS	Diagnosed without CBDS	*p*value
*Age*					
<75	398 (398/466)	58 ± 14.50	259 (259/398)	139 (139/398)	0.007
≥75	68 (68/466)		56 (56/68)	12 (12/68)	

*Gender*					
Male	198 (198/466)	—	149 (149/198)	49 (49/198)	0.002
Female	268 (268/466)		166 (166/268)	102 (102/268)	

*Surgical procedure*					
LC + LTCBDE	448 (448/466)		297 (297/448)	151 (151/448)	—
Non-lc + LTCBED	18 (18/466)		18 (100)	0 (zero)	

*Preoperative MRCP*					
Positive	181 (181/349)	—	169 (169/349)	12 (12/349)	<0.0001
Negative	168 (168/349)		83 (83/349)	85 (85/349)	

*Preoperative common bile duct imaging width*					
<0.8 cm	242 (242/250)	0.8 ± 0.4	0.56 ± 0.10	0.54 ± 0.09	<0.0001
≥0.8 cm	208 (208/250)		1.11 ± 0.35	0.93 ± 0.18	

*Preoperative biochemical indicators*					
ALT	466 (100)	52.7 ± 94.7	65.57 ± 110.35	25.78 ± 34.39	<0.0001
AST		34.6 ± 53.4	41.12 ± 63.28	20.86 ± 13.52	<0.0001
ALP		122.5 ± 97.5	141.44 ± 112.10	82.84 ± 28.33	<0.0001
GGT		141.5 ± 227.5	185.40 ± 262.21	50.02 ± 62.15	<0.0001
TB		21.1 ± 30.1	25.26 ± 41.54	14.35 ± 7.52	0.001
DB		7.9 ± 18.2	10.49 ± 25.17	2.97 ± 2.37	<0.0001

**Table 2:** The diagnostic efficacy of the predictors for common bile duct in all patients.

Variable (s)	Sen	Spe	AUC	SE	95% confidence interval	*p*
Age + gender	79.37	40.4	61.7	0.0275	0.571∼0.661	<0.0001
ALT	72.06	58.28	70.3	0.0248	0.659∼0.744	<0.0001
AST	60.63	66.89	67.8	0.0256	0.634∼0.720	<0.0001
ALP	60	85.43	0.753	0.0225	0.711∼0.791	<0.0001
TB	39.49	86.75	66.3	0.0258	0.618∼0.706	<0.0001
DB	47.13	86.75	70	0.0244	0.656∼0.742	<0.0001
GGT	78.1	63.58	76.1	0.0225	0.720∼0.799	<0.0001
CBDD	56.77	82.99	74.7	0.0233	0.704∼0.786	<0.0001
MRCP	70.63	87.63	80.4	0.0261	0.759∼0.845	<0.0001
Total	76.11	86.6	87.2	0.02	0.832∼0.906	<0.0001

**Table 3:** The diagnostic efficacy of the predictors for common bile duct in patients with negative result of MRCP.

Variable (s)	Sen	Spe	AUC	SE	95% confidence interval	*p*
Age + gender	38.55	82.35	60.7	0.0439	0.529∼0.681	0.015
ALT	66.27	60.00	65.4	0.0422	0.577∼0.725	0.0003
AST	57.83	67.06	62.8	0.0432	0.550∼0.701	0.003
ALP	55.42	85.88	70.1	0.0411	0.626∼0.769	<0.0001
TB	45.78	84.71	63.0	0.0437	0.553∼0.704	0.0028
DB	55.42	76.47	65.2	0.0428	0.574∼0.723	0.0004
GGT	69.88	68.24	70.4	0.0407	0.629∼0.772	<0.0001
CBDD	39.27	90.59	63.8	0.0433	0.560∼0.711	0.0014
Total	56.79	88.24	75.9	0.0377	0.687∼0.822	<0.0001

**Table 4:** The diagnostic efficacy of the predictors for common bile duct in patients with both negative results of MRCP and CBDD.

Variable (s)	Sen	Spe	AUC	SE	95% Confidence interval	*p*
Age + Gender	65.52	57.89	59	0.0508	0.502∼0.674	0.0753
ALT	50	75	65.8	0.474	0.571∼0.738	0.0009
AST	72.41	47.37	61.5	0.049	0.527∼0.698	0.0189
ALP	63.79	73.68	70.9	0.0468	0.624∼0.784	<0.0001
TB	68.97	56.58	60.1	0.0499	0.513∼0.685	0.0425
DB	84.48	48.68	65	0.0483	0.562∼0.730	0.0019
GGT	65.52	68.42	71.5	0.0453	0.630∼0.789	<0.0001
Total	72.41	69.74	73.2	0.0455	0.649∼0.805	<0.0001

## Data Availability

All the medical records used in this retrospective clinical study were authentic and reliable, and the data collection process was supervised by the Ethics Committee of Beijing Friendship Hospital. All readers may request access to the original data and medical records by e-mail to the corresponding author.
